# Exploring the Antiovarian Cancer Mechanisms of Salvia Miltiorrhiza Bunge by Network Pharmacological Analysis and Molecular Docking

**DOI:** 10.1155/2022/7895246

**Published:** 2022-11-29

**Authors:** Xiao Xu, Zhiwei Zhang, Likun Liu, Cheng Che, Weiling Li

**Affiliations:** ^1^Department of Biotechnology, Dalian Medical University, Dalian, China; ^2^Division of Regulatory Glycobiology, Institute of Molecular Biomembrane and Glycobiology, Tohoku Medical and Pharmaceutical University, Sendai, Japan; ^3^Medical Imaging Diagnosis Centre, General Hospital of Fushun Mining Bureau of Liaoning Health Industry Group, Fushun, China; ^4^Liaoning Key Laboratory of Hematopoietic Stem Cell Transplantation and Translational Medicine, Second Hospital of Dalian Medical University, Dalian, China

## Abstract

**Background:**

Ovarian cancer was one of the gynecological malignant tumors. *Salvia miltiorrhiza* Bunge (SMB) was a kind of herbal medicine with an antitumor effect. However, the inhibitory effect of SMB on ovarian cancer and its potential mechanism were still unclear.

**Objective:**

The antitumor effect of SMB on ovarian cancer was studied by network pharmacology and molecular docking techniques, and its possible molecular mechanisms were analyzed.

**Method:**

The active ingredients of SMB and the target data of ovarian cancer were obtained from the Traditional Chinese Medicines for Systems Pharmacology Database (TCMSP) and the GeneCards database. The relationship between active ingredients of SMB and ovarian cancer targets was analyzed by String database, David 6.8 online database, and Cytoscape 3.7.2 software, and then potential pathways were screened out. In addition, molecular docking technology was used to verify further the binding effect of antiovarian cancer pathway targets with active ingredients of SMB. Finally, survival analysis was performed for all potential targets.

**Results:**

We analyzed 71 SMB–ovarian cancer common targets, and the Kyoto Encyclopedia of Genes and Genomes (KEGG) enrichment analysis showed that the PI3K-Akt signaling pathway might be an essential pathway for SMB to inhibit ovarian cancer. Luteolin, Tanshinone IIA, and Cryptotanshinone in SMB might play an important role. HSP90AA1, CDK2, and PIK3CG might be potential targets of SMB in inhibiting ovarian cancer.

**Conclusion:**

Through network pharmacology and molecular docking analysis, we found that SMB might partially inhibit ovarian cancer by the PI3K-Akt signaling pathway. We believe that SMB might be a potential therapeutic agent for ovarian cancer patients.

## 1. Introduction

Ovarian cancer was one of the most common malignancies of the female reproductive organs [1]. Because ovarian cancer was located in the deep pelvic cavity, had a small volume, and had no apparent symptoms, the early diagnosis of ovarian cancer was challenging, the mortality rate was very high, and it was a severe threat to women's health [2]. The treatment of ovarian cancer mainly included surgery and using taxane and platinum chemotherapeutic agents [3], but these drugs had toxic side effects. However, the treatment prognosis was poor [4]. Therefore, it was necessary to explore more safe ovarian cancer drugs with good prognosis.

Studies have shown that traditional Chinese medicine (TCM) could inhibit the proliferation and metastasis of tumor cells because of its low toxicity, and it was widely used [5]. *Salvia miltiorrhiza* Bunge (SMB) was the dried root and rhizome of the *Lamiaceae* plant, a TCM. It has been widely used in traditional medicine for a long time, showing a variety of biological activities in clinical practice, such as antioxidative stress, antiplatelet aggregation, and anti-inflammatory effects [6]. More importantly, SMB has a good anticancer effect and great potential in cancer treatment, and it was widely used in treating cancer in TCM [7]. It has been proved that SMB could inhibit breast cancer [8], liver cancer [9], stomach cancer [10], and nonsmall cell lung cancer [11]. Our study investigated the antiovarian cancer effect and potential molecular mechanisms of SMB.

Network pharmacology combined drug targets with human disease genes, effectively elucidating the mechanism of action of the drugs and efficiently screening drugs [12]. Network pharmacology improved patient outcomes by integrating multiple disciplines such as bioinformatics, systems biology, and multivariate pharmacology to provide better treatment options and understand the side effects of drugs [13]. In 2011, Li proposed the concept of network pharmacology of TCM. It combines network pharmacology with TCM, providing new ideas for treating diseases and revealing the mechanism of action of drugs and their potential to predict the active ingredients of drugs and to determine their mechanism of action [14]. In recent years, molecular docking technology has been essential in exploring affinity binding sites between drug-active ingredients and disease targets [15].

In this study, network pharmacology and molecular docking techniques were used to explore the active ingredients and specific molecular mechanisms of SMB in ovarian cancer. We found that SMB might inhibit the development of ovarian cancer mainly by acting on the PI3K-Akt signaling pathway. Luteolin, Tanshinone IIA, and Cryptotanshinone might be the essential antitumor active ingredients in SMB; however, the synergistic effect of other components could not be excluded. This study pointed the way for the further application of SMB in treating ovarian cancer.

## 2. Materials and Methods

### 2.1. Data Preparation

Downloaded SMB active ingredient data from the online database: the Traditional Chinese Medicines for Systems Pharmacology Database [16] (TCMSP, https://tcmspw.com/tcmsp.php). Screening conditions were set as drug-likeness (DL) ≥ 0.18 and oral bioavailability (OB) ≥ 30%. The target genes and the MOL2 file of the 3D structure of active ingredients could be obtained from this website. PyMOL software [17] was used to convert MOL2 files to PDB files.

Downloaded ovarian cancer disease target genes from the GeneCards database [18] (https://www.genecards.org).Among the SMB ingredient target genes and ovarian cancer genes, there were some identical genes with mismatched names, and the names of these genes were unified by using the UniProt [19] (https://www.uniprot.org). Downloaded the PDB file of the gene receptor protein online from the RCSB PDB website [20] (http://www.rcsb.org/).

### 2.2. Network Pharmacology

Venn maps of SMB and ovarian cancer targets were plotted online on the Jvenn website (http://www.bioinformatics.com.cn/static/others/jvenn/), and the data of common targets of SMB and ovarian cancer were obtained. The protein-protein interaction (PPI) data was analyzed on STRING [21] (https://string-db.org).

The enrichment analysis of the shared genes of SMB and ovarian cancer was performed on the DAVID Bioinformatics Resources 6.8 [22] (https://david.ncifcrf.gov). The data from the Kyoto Encyclopedia of Genes and Genomes (KEGG), Cellular Component (CC), Biological Process (BP), and Molecular Function (MF) obtained were plotted on the Ehbio (http://www.ehbio.com/) website.

Cytoscape 3.7.2 [23] software was used to visualize the PPI, SMB active ingredients, common targets of drug diseases, and the relationship between targets in the pathway and their corresponding active ingredients. The nodes were arranged according to the degree value from the largest to the smallest. The number of connecting lines between the target and the active ingredient was proportional to the correlation between the target and the active ingredient.

### 2.3. Molecular Docking Technology

AutoDockTools 1.5.6 [24] software was used to modify the protein PDB file, including removal of ligands and water, hydrogenation, amino acid optimization, and repair and set the parameters of the docking site of the receptor protein, including the active sites to which the small molecule ligand might bind. The modified receptor protein and ligand small molecule PDBQT files were generated. The protein receptor was docked with the small molecule ligand, and the binding energy was calculated.

### 2.4. Survival Analysis

The survival analysis of common target genes of SMB–ovarian cancer was analyzed online on the GEPIA website [25] (http://gepia.cancer-pku.cn/); the site contains RNA sequencing expression data from 9,736 tumors and 8,587 normal samples from the TCGA and GTEX projects. The conditions of analysis were as follows: Methods–Overall Survival; Group Cutoff–Median; Datasets Selection–OV. Keep data with *P* < 0.05. Relationships between genes of interest in survival analysis and their associated active ingredients were presented by Cytoscape 3.7.2 software.

## 3. Results

### 3.1. Screening of Active Ingredients and Targets of SMB

The active ingredients data of SMB was downloaded from the TCMSP website, and the screening value was set as DL ≥ 0.18 and OB ≥ 30%. 65 active ingredients were screened and obtained, corresponding to 137 action targets (Table 1).

### 3.2. “SMB–Ovarian Cancer” Target Data Analysis

The GeneCards database obtained 7070 ovarian cancer-related targets, and the correlation score of screening criteria was ≥15. Finally, we obtained 1118 qualified targets. Among them, 71 targets were the common targets of ovarian cancer and SMB, which were the focus of our subsequent analysis (Figure 1(a)).

### 3.3. “SMB–Ovarian Cancer” Targets Network

The interaction between SMB–Ovarian Cancer common target proteins was analyzed in the String online database, and 1168 edges were obtained (Figure 1(b)). The top five targets were TP53 (Tumor Protein P53), AKT1 (AKT Serine/Threonine Kinase 1), MAPK1 (Mitogen-Activated Protein Kinase 1), VEGFA (Vascular Endothelial Growth Factor A), and EGFR (Epidermal Growth Factor Receptor).

We used the software Cytoscape 3.7.2 to analyze the relationship between the common target of “SMB–Ovarian” and the active ingredients of SMB (Figure 1(c)). We had 71 target nodes, 58 active ingredient nodes, and 332 edges. The degree value of the node decreased with the correlation, which was reflected by the size. The top three targets were PTGS2 (Prostaglandin-Endoperoxide Synthase 2), F2 (Coagulation Factor II, Thrombin), and PTGS1 (Prostaglandin-Endoperoxide Synthase 1); active ingredients were Luteolin, Tanshinone IIA, and dan-shexinkum d. The results showed that the active ingredients of SMB could closely bind to some of the pathogenic targets of ovarian cancer.

### 3.4. Enrichment Analysis

The data of SMB–Ovarian Cancer common targets were uploaded to the David website for KEGG and GO enrichment analyses, and data results of *P* < 0.01 was retained: 196 GO-BP results, 23 GO-CC results, 47 GO-MF results, and 91 KEGG results. We listed the top 10 GO-BP, GO-CC, GO-MF, and 15 pathways strongly associated with ovarian cancer (Figure 2) (Table 2). In the KEGG enrichment diagram, the PI3K-Akt signaling pathway showed a strong correlation, which was much higher than other pathways. We hypothesized that SMB might have an inhibitory effect on ovarian cancer mainly through the PI3K-Akt signaling pathway.

### 3.5. PI3K-Akt Signaling Pathway Played an Important Role in the Inhibition of Ovarian Cancer by SMB

The relationship between target genes in the PI3K-Akt signaling pathway and active ingredients of SMB was further analyzed. 25 targets in the PI3K-Akt signaling pathway could bind to 32 active ingredients in SMB. Among them, the top ten were: HSP90AA1 (Heat Shock Protein 90 Alpha Family Class A Member 1), PIK3CG (Phosphatidylinositol-4,5-Bisphosphate 3-Kinase Catalytic Subunit Gamma), CDK2 (Cyclin Dependent Kinase 2), GSK3B (Glycogen Synthase Kinase 3 Beta), RELA (RELA Proto-Oncogene, NF-KB Subunit), TP53, CDKN1A (Cyclin Dependent Kinase Inhibitor 1A), BCL2L1 (BCL2 Like 1), CCND1 (Cyclin D1), and IL2 (Interleukin 2). The top three active ingredients were Luteolin, Tanshinone IIA, and Neocryptotanshinone II, a total of 73 stably bound combinations (Figure 3(a)). To further verify whether the active ingredients of SMB can effectively bind to the target of the PI3K-Akt signaling pathway. We selected the top ten target genes and active ingredients for molecular docking. We then obtained 30 groups of molecular docking results and their binding energy (The smaller the binding energy, the more stable the binding.) (Figure 3(b)) (Table 3). The binding energies of HSP90AA1, PIK3CG, CDK2, and GSK3B with active ingredients were generally low, indicating that their binding was more stable. Among the active components, Neocryptotanshinone II, Cryptotanshinone, 1-methyl-8,9-dihydro-7H-naphtho [5,6-g] benzofuran-6,10,11-trione, miltionone I, Isotanshinone II, epidanshenspiroketallactone, and dihydrotanshinoneI were more stable in binding to target proteins. The results demonstrated that the SMB's active ingredients could affect the growth of ovarian cancer cells by acting on targets in the PI3K-Akt signaling pathway.

### 3.6. Survival Analysis

We analyzed the survival of 71 common genes in the TCGA database in ovarian cancer patients. Nine genes that were closely related to the prognosis of ovarian cancer patients were screened, as follows: IFNG (Interferon Gamma), BIRC5 (Baculoviral IAP Repeat Containing 5), MMP1 (Matrix Metallopeptidase 1), ERBB2 (Erb-B2 Receptor Tyrosine Kinase 2), RB1 (RB Transcriptional Corepressor 1), MYC (MYC Proto-Oncogene, BHLH Transcription Factor), BCL2L1, CD40LG (CD40 Ligand), and PTPN1 (Protein Tyrosine Phosphatase NonReceptor Type 1) (Figure 4(a)). The difference in the expression of these genes would significantly impact the prognosis of ovarian cancer patients. By analyzing the relationships between the nine target genes and the active ingredients of SMB, we found that Luteolin and Cryptotanshinone had essential effects on the survival of patients (Figure 4(b)). The results showed that the active ingredients of SMB not only effectively inhibit the development of ovarian cancer but also affect the prognosis and survival of ovarian cancer patients.

## 4. Discussion

In advanced cases of ovarian cancer, the most lethal cancer of the female reproductive system, the five-year survival rate was less than 30 percent [4]. In order to avoid the toxic side as much as possible and improve patients' quality of life, many cases of treating ovarian cancer with the active ingredients of TCM have emerged in recent years [26, 27]. SMB was a traditional Chinese herb once widely used to treat various diseases. In recent years, there have been some reports on the inhibitory effect of SMB on cancer, such as breast cancer [28, 29], prostate cancer [30], oral cancer [31], and other tumors [32]. Our study explored the potential mechanism of effective ingredients of SMB against ovarian cancer through network pharmacological methods and molecular docking techniques.

Through network pharmacology, molecular docking techniques, and survival analysis, we obtained a systematic evaluation of the active ingredients of SMB. Luteolin and Tanshinone IIA showed high value in analyzing the relationship between SMB and ovarian cancer, the analysis of the relationship between the PI3K-Akt signaling pathway and SMB, and the analysis of patients' survival. Luteolin had been reported to inhibit ovarian cancer metastasis by downregulating MMP2 (Matrix Metallopeptidase 2) and MMP9 (Matrix Metallopeptidase 9) [33]. Cell experiments proved that Luteolin had an inhibitory effect on the growth of ovarian cancer cells [34, 35]. In our study, the impact of Luteolin involved multiple genes of the PI3K-Akt signaling pathway and related to survival. Tanshinone IIA inhibited ovarian cancer growth by inhibiting the PI3K/AKT/JNK signaling pathway, malignant properties, and angiogenesis [36, 37]. Cryptotanshinone showed good performance in survival analysis and the analysis of the relationship between the PI3K-Akt signaling pathway and SMB and showed a relatively good binding effect in molecular docking results [38, 39]. We speculated that Luteolin, Tanshinone IIA, and Cryptotanshinone might play essential roles in inhibiting ovarian cancer by SMB. However, we could not exclude other remaining active ingredients that were equally important and cooperative throughout the process. Whether the combination of different components can get a better inhibitory effect is also the focus of our future research.

In KEGG enrichment analysis, the PI3K-Akt signaling pathway stood out among many pathways. The PI3K-Akt signaling pathway played a crucial role in tumors' malignant transformation, growth, proliferation, and metastasis. Different levels of genetic aberrations in the PI3K pathway were often observed in ovarian cancer, leading to overactivation of the pathway [40]. Many PI3K/Akt/mTOR pathway inhibitors for ovarian cancer have been reported in preclinical and clinical data [41]. Previous studies by our group had confirmed that Dihydrotanshinone I, an essential ingredient in SMB, could inhibit the proliferation and migration of ovarian cancer cells in vitro and in vivo by regulating the PI3K/Akt signaling pathway [42]. The study by Deng et al. also believed that the PI3K-Akt signaling pathway was an essential pathway for compound *Salvia miltiorrhiza* drugs to act on ovarian cancer [43]. In our research results, the PI3K-Akt signaling pathway could stably bind to the active components of SMB, and the molecular docking results also agreed with our previous results. Thus, we believe that SMB inhibits ovarian cancer proliferation by affecting the PI3K-Akt signaling pathway. Of course, more experiments are needed to explore the relationship between the PI3K-Akt signaling pathway and SMB's critical active ingredients in ovarian cancer to verify our view further.

HSP90AA1 and CDK2 were selected by the analysis of the relationship between SMB and ovarian cancer, and the relationship between the PI3K-Akt signaling pathway and SMB. The molecular docking showed that they could stably bind to the active ingredients of SMB. Abnormal expression of HSP90AA1 and CDK2 could affect the progression of ovarian cancer [44, 45]. PIK3CG was the second target gene in the analysis of the interaction between the PI3K-Akt signaling pathway and the active ingredients of SMB, and it had a high molecular docking score. Zhang et al. suggested that it might be a potential therapeutic target for epithelial ovarian cancer [46]. PTPN1 was associated with multiple active ingredients of SMB in survival analysis; studies had shown that the overexpression of PTPN1 in high-grade serous carcinoma might be a marker of better response to chemotherapy [47]. These results suggested that SMB might inhibit ovarian cancer by acting on PTPN1. HSP90AA1, CDK2, and PIK3CG belong to the PI3K-Akt signaling pathway.

## 5. Conclusions

In conclusion, based on network pharmacology and molecular docking analysis, we believe that Luteolin, Tanshinone IIA, and Cryptotanshinone might be the main active ingredients of SMB in inhibiting ovarian cancer because they act on a lot of ovarian cancer genes. In addition, the PI3K-Akt signaling pathway might be the main pathway for SMB to inhibit ovarian cancer because the significant genes HSP90AA1, CDK2, and PIK3CG in this pathway receive the action of multiple ingredients in SMB. However, the synergistic effect of various ingredients were more critical in herbal compounds. This study was conducted to explore the therapeutic potential of SMB further and analyzed the action mechanism of active ingredients in SMB. It allows for applying SMB as a new Chinese herbal therapy in treating ovarian cancer.

## Figures and Tables

**Figure 1:** Screening of common targets between SMB and ovarian cancer. (a) 1118 ovarian cancer targets intersected137 SMB targets for 71 common targets. (b) Common targets protein-protein interaction (PPI) network. (c) Relationship between SMB active ingredients and the SMB–ovarian cancer common targets. Green-ingredient; Blue-target.

**Figure 2:** Analysis of enrichment. (a) The top ten of GO-BP, GO-CC, and GO-MF enrichment. (b) 15 KEGG pathways that were highly correlated with ovarian cancer.

**Figure 3:** Relationship between the PI3K-Akt signaling pathway and active ingredients. (a) Relationship between targets in the PI3K-Akt signaling pathway and active ingredients in SMB. Green-ingredient; Blue-target. (b) Molecular docking results between representative SMB active ingredients and the PI3K-Akt signaling pathway targets.

**Figure 4:** Survival analysis. (a) Survival analysis of SMB-ovarian cancer common targets (*P* < 0.05). (b) Relationship between significant genes in survival analysis and active ingredients of SMB. Green-ingredient; Blue-target.

**Table 1:** Major active ingredients of SMB.

Mol ID	Molecule name	OB (%)	DL	Target
MOL001601	1,2,5,6-tetrahydrotanshinone	38.75	0.36	29
MOL001659	Poriferasterol	43.83	0.76	2
MOL001771	Poriferast-5-en-3beta-ol	36.91	0.75	2
MOL001942	Isoimperatorin	45.46	0.23	1
MOL002222	Sugiol	36.11	0.28	17
MOL002651	Dehydrotanshinone II A	43.76	0.4	21
MOL002776	Baicalin	40.12	0.75	2
MOL000569	Digallate	61.85	0.26	3
MOL000006	Luteolin	36.16	0.25	57
MOL006824	*α*-Amyrin	39.51	0.76	0
MOL007036	5,6-dihydroxy-7-isopropyl-1,1-dimethyl-2,3-dihydrophenanthren-4-one	33.77	0.29	17
MOL007041	2-isopropyl-8-methylphenanthrene-3,4-dione	40.86	0.23	33
MOL007045	3*α*-hydroxytanshinoneIIa	44.93	0.44	13
MOL007048	(E)-3-[2-(3,4-dihydroxyphenyl)-7-hydroxy-benzofuran-4-yl]acrylic acid	48.24	0.31	3
MOL007049	4-methylenemiltirone	34.35	0.23	33
MOL007050	2-(4-hydroxy-3-methoxyphenyl)-5-(3-hydroxypropyl)-7-methoxy-3-benzofurancarboxaldehyde	62.78	0.4	12
MOL007051	6-o-syringyl-8-o-acetyl shanzhiside methyl ester	46.69	0.71	0
MOL007058	Formyltanshinone	73.44	0.42	8
MOL007059	3-beta-Hydroxymethyllenetanshiquinone	32.16	0.41	17
MOL007061	Methylenetanshinquinone	37.07	0.36	24
MOL007063	Przewalskin a	37.11	0.65	2
MOL007064	Przewalskin b	110.32	0.44	6
MOL007068	Przewaquinone B	62.24	0.41	9
MOL007069	Przewaquinone c	55.74	0.4	22
MOL007070	(6S,7R)-6,7-dihydroxy-1,6-dimethyl-8,9-dihydro-7H-naphtho[8,7-g]benzofuran-10,11-dione	41.31	0.45	8
MOL007071	Przewaquinone f	40.31	0.46	5
MOL007077	Sclareol	43.67	0.21	1
MOL007079	Tanshinaldehyde	52.47	0.45	13
MOL007081	Danshenol B	57.95	0.56	8
MOL007082	Danshenol A	56.97	0.52	9
MOL007085	Salvilenone	30.38	0.38	8
MOL007088	Cryptotanshinone	52.34	0.4	30
MOL007093	Dan-shexinkum d	38.88	0.55	29
MOL007094	Danshenspiroketallactone	50.43	0.31	25
MOL007098	Deoxyneocryptotanshinone	49.4	0.29	28
MOL007100	Dihydrotanshinlactone	38.68	0.32	36
MOL007101	dihydrotanshinoneI	45.04	0.36	17
MOL007105	Epidanshenspiroketallactone	68.27	0.31	26
MOL007107	C09092	36.07	0.25	12
MOL007108	Isocryptotanshi-none	54.98	0.39	31
MOL007111	Isotanshinone II	49.92	0.4	26
MOL007115	Manool	45.04	0.2	1
MOL007118	Microstegiol	39.61	0.28	0
MOL007119	Miltionone I	49.68	0.32	28
MOL007120	Miltionone II	71.03	0.44	8
MOL007121	Miltipolone	36.56	0.37	2
MOL007122	Miltirone	38.76	0.25	26
MOL007123	Miltirone II	44.95	0.24	0
MOL007124	Neocryptotanshinone ii	39.46	0.23	29
MOL007125	Neocryptotanshinone	52.49	0.32	16
MOL007127	1-methyl-8,9-dihydro-7H-naphtho[5,6-g]benzofuran-6,10,11-trione	34.72	0.37	20
MOL007130	Prolithospermic acid	64.37	0.31	10
MOL007132	(2R)-3-(3,4-dihydroxyphenyl)-2-[(Z)-3-(3,4-dihydroxyphenyl)acryloyl]oxy-propionic acid	109.38	0.35	8
MOL007140	(Z)-3-[2-[(E)-2-(3,4-dihydroxyphenyl)vinyl]-3,4-dihydroxy-phenyl]acrylic acid	88.54	0.26	0
MOL007141	Salvianolic acid g	45.56	0.61	1
MOL007142	Salvianolic acid j	43.38	0.72	3
MOL007143	Salvilenone I	32.43	0.23	8
MOL007145	Salviolone	31.72	0.24	38
MOL007149	NSC 122421	34.49	0.28	0
MOL007150	(6S)-6-hydroxy-1-methyl-6-methylol-8,9-dihydro-7H-naphtho[8,7-g]benzofuran-10,11-quinone	75.39	0.46	8
MOL007151	Tanshindiol B	42.67	0.45	7
MOL007152	Przewaquinone E	42.85	0.45	7
MOL007154	Tanshinone iia	49.89	0.4	41
MOL007155	(6S)-6-(hydroxymethyl)-1,6-dimethyl-8,9-dihydro-7H-naphtho[8,7-g]benzofuran-10,11-dione	65.26	0.45	13
MOL007156	Tanshinone VI	45.64	0.3	13

65 major active ingredients in *Salvia miltiorrhiza* and the number of ovarian cancer targets corresponding to each ingredient.

**Table 2:** KEGG pathways.

No	Term	*P* Value	Genes
1	PI3K-Akt signaling pathway	5.88E-15	GSK3B, CDKN1A, ITGB3, RELA, EGFR, PIK3CG, CASP9, CCND1, MYC, AKT1, MAPK1, MCL1, HSP90AA1, INSR, IL2, VEGFA, IL4, IL6, CDK4, CDK2, BCL2, MDM2, MET, TP53, and BCL2L1

2	T cell receptor signaling pathway	2.19E-14	IL10, GSK3B, JUN, FOS, MAPK14, TNF, IL2, PIK3CG, RELA, IL4, NFKBIA, CD40LG, IFNG, CDK4, AKT1, and MAPK1

3	TNF signaling pathway	6.21E-14	JUN, EDN1, FOS, PTGS2, MAPK14, TNF, MMP9, PIK3CG, RELA, ICAM1, NFKBIA, CASP7, IL6, CASP3, AKT1, and MAPK1

4	HIF-1 signaling pathway	2.67E-13	CDKN1A, EDN1, NOS2, INSR, STAT3, EGFR, PIK3CG, RELA, VEGFA, IL6, IFNG, ERBB2, BCL2, AKT1, and MAPK1

5	Apoptosis	1.30E-11	NFKBIA, CASP9, CASP7, CASP3, BCL2, XIAP, AKT1, TNF, TP53, RELA, PIK3CG, and BCL2L1

6	Viral carcinogenesis	8.09E-11	RB1, CDKN1A, JUN, STAT3, PIK3CG, RELA, NFKBIA, CCNA2, CCND1, CDK4, CASP3, CHEK1, CDK2, MDM2, MAPK1, PRKACA, and TP53

7	FoxO signaling pathway	4.08E-10	IL10, CDKN1A, INSR, STAT3, MAPK14, EGFR, PIK3CG, IL6, CCNB1, CCND1, CDK2, MDM2, AKT1, and MAPK1

8	Prolactin signaling pathway	1.29E-09	GSK3B, CCND1, STAT3, MAPK1, AKT1, FOS, MAPK14, ESR1, RELA, ESR2, and PIK3CG

9	Cell cycle	2.1E-09	RB1, GSK3B, CDKN1A, PCNA, CCNA2, CCNB1, CCND1, CDK4, MYC, CHEK1, CDK2, MDM2, and TP53

10	Estrogen signaling pathway	2.4E-09	HSP90AA1, JUN, MMP2, MAPK1, AKT1, FOS, PRKACA, ESR1, MMP9, EGFR, ESR2, and PIK3CG

11	Thyroid hormone signaling pathway	1.2E-08	CASP9, GSK3B, CCND1, MYC, ITGB3, MDM2, MAPK1, AKT1, PRKACA, ESR1, TP53, and PIK3CG

12	p53 signaling pathway	1.4E-08	CASP9, CDKN1A, CCNB1, CCND1, CDK4, CASP3, CHEK1, CDK2, MDM2, and TP53

13	MicroRNAs in cancer	8.1E-08	CDKN1A, ITGB3, STAT3, PTGS2, MMP9, EGFR, VEGFA, CCND1, MYC, CASP3, ERBB2, MDM2, BCL2, MET, TP53, and MCL1

14	Focal adhesion	6.3E-07	GSK3B, JUN, ITGB3, XIAP, EGFR, PIK3CG, VEGFA, CCND1, ERBB2, BCL2, AKT1, MAPK1, and MET

15	Toll-like receptor signaling pathway	8.048E-07	NFKBIA, IL6, JUN, MAPK1, AKT1, FOS, MAPK14, TNF, RELA, and PIK3CG

15 KEGG pathways that were highly correlated with ovarian cancer. The pathways were arranged according to *P* Values, and the genes contained in the pathways were listed.

**Table 3:** Molecular docking results.

Target name	PDB ID	Compound	Mol ID	Binding energy
HSP90AA1	5FWK	1-methyl-8,9-dihydro-7H-naphtho[5,6-g]benzofuran-6,10,11-trione	MOL007127	-7.11
HSP90AA1	5FWK	Epidanshenspiroketallactone	MOL007105	-6.88
HSP90AA1	5FWK	dihydrotanshinoneI	MOL007101	-6.57
HSP90AA1	5FWK	Neocryptotanshinone ii	MOL007124	-5.87
HSP90AA1	5FWK	Luteolin	MOL000006	-4.54
HSP90AA1	5FWK	2-(4-hydroxy-3-methoxyphenyl)-5-(3-hydroxypropyl)-7-methoxy-3-benzofurancarboxaldehyde	MOL007050	-4.12
PIK3CG	2A4Z	1-methyl-8,9-dihydro-7H-naphtho[5,6-g]benzofuran-6,10,11-trione	MOL007127	-7.99
PIK3CG	2A4Z	dihydrotanshinoneI	MOL007101	-7.78
PIK3CG	2A4Z	Luteolin	MOL000006	-6.51
CDK2	2CCH	Epidanshenspiroketallactone	MOL007105	-8.35
CDK2	2CCH	Neocryptotanshinone ii	MOL007124	-7.89
CDK2	2CCH	Miltionone I	MOL007119	-7.42
CDK2	2CCH	Isotanshinone II	MOL007111	-7.28
CDK2	2CCH	2-(4-hydroxy-3-methoxyphenyl)-5-(3-hydroxypropyl)-7-methoxy-3-benzofurancarboxaldehyde	MOL007050	-4.36
GSK3B	4AFJ	Miltionone I	MOL007119	-6.77
GSK3B	4AFJ	Isotanshinone II	MOL007111	-6.7
GSK3B	4AFJ	Neocryptotanshinone ii	MOL007124	-6.32
GSK3B	4AFJ	2-(4-hydroxy-3-methoxyphenyl)-5-(3-hydroxypropyl)-7-methoxy-3-benzofurancarboxaldehyde	MOL007050	-4
RELA	1NFI	Cryptotanshinone	MOL007088	-7.06
RELA	1NFI	Tanshinone iia	MOL007154	-6.44
RELA	1NFI	Luteolin	MOL000006	-5.59
TP53	2K8F	Tanshinone iia	MOL007154	-5.4
TP53	2K8F	Luteolin	MOL000006	-3.75
CDKN1A	2ZVW	Tanshinone iia	MOL007154	-5.71
CDKN1A	2ZVW	Luteolin	MOL000006	-4.63
BCL2L1	4CIN	Cryptotanshinone	MOL007088	-6.12
BCL2L1	4CIN	Luteolin	MOL000006	-3.89
CCND1	2 W96	Cryptotanshinone	MOL007088	-7.56
CCND1	2 W96	Luteolin	MOL000006	-4.93
IL2	7AH1	Luteolin	MOL000006	-4.38

Molecular docking results between representative SMB active ingredients and the PI3K-Akt signaling pathway targets. And it listed the binding energy.

## Data Availability

The network pharmacology and molecular docking data used to support the findings of this study are available from the corresponding author upon request.
